RETRACTED

# A β-Lactamase Based Reporter System for ESX Dependent Protein Translocation in Mycobacteria

**DOI:** 10.1371/journal.pone.0035453

**Published:** 2012-04-18

**Authors:** Tobias Rosenberger, Juliane K. Brülle, Peter Sander

**Affiliations:** 1 Institute of Medical Microbiology, University of Zurich, Zurich, Switzerland; 2 Nationales Zentrum für Mykobakterien, Zurich, Switzerland; French National Centre for Scientific Research - Université de Toulouse, France

## Abstract

Protein secretion is essential for all bacteria in order to interact with their environment. *Mycobacterium tuberculosis* depends on protein secretion to subvert host immune response mechanisms. Both the general secretion system (Sec) and the twin-arginine translocation system (Tat) are functional in mycobacteria. Furthermore, a novel type of protein translocation system named ESX has been identified. In the genome of *M. tuberculosis* five paralogous ESX regions (ESX-1 to ESX-5) have been found. Several components of the ESX translocation apparatus have been identified over the last ten years. The ESX regions are composed of a basic set of genes for the translocation machinery and the main substrate - a heterodimer. The best studied of these heterodimers is EsxA (ESAT-6)/EsxB (CFP-10), which has been shown to be exported by ESX-1. EsxA/B is heavily involved in virulence of *M. tuberculosis*. EsxG/H is exported by ESX-3 and seems to be involved in an essential iron-uptake mechanism in *M. tuberculosis*. These findings make ESX-3 components high profile drug targets. Until now, reporter systems for determination of ESX protein translocation have not been developed. In order to create such a reporter system, a truncated β-lactamase (‘*bla TEM*-1) was fused to the N-terminus of EsxB, EsxG and EsxU, respectively. These constructs have then been tested in a β-lactamase (BlaS) deletion strain of *Mycobacterium smegmatis*. *M. smegmatis* Δ*blaS* is highly susceptible to ampicillin. An ampicillin resistant phenotype was conferred by translocation of Bla TEM-1-Esx fusion proteins into the periplasm. BlaTEM-1-Esx fusion proteins were not found in the culture filtrate suggesting that plasma membrane translocation and outer membrane translocation are two distinct steps in ESX secretion. Thus we have developed a powerful tool to dissect the molecular mechanisms of ESX dependent protein translocation and to screen for novel components of the ESX systems on a large scale.

## Introduction

Tuberculosis (TB) is a chronic, contagious disease caused by several members of the *Mycobacterium tuberculosis* complex [1]. Although marginalized in America and central Europe, TB remains an overwhelming burden on humanity. Approx. 2 billion people - about a third of the world's population - are carrier of the pathogen, making TB a pandemic. Among these people, 5–10% develop symptoms and become infectious themselves [2]. An estimated 1.7 million infected people die from TB every year.

RETRACTED

Subversion of the normal progression of the phagosomal compartment into an active, bactericidal lysosomal compartment is one of the key features of *M. tuberculosis* pathogenicity [3], [4]. As an additional resistance factor, mycobacteria possess a nearly impenetrable cell envelope which protects the bacteria against physical and chemical stress. This cell envelope also plays a crucial role in intrinsic drug resistance in pathogenic mycobacteria, and is one of the key features of persistence in latency [5]. The unique mycobacterial cell envelope consists of a phospholipid bilayer plasma membrane (PM), followed by a periplasmatic space (PP) with two electron dense layers of unconfirmed identity [6]. The inner of these layers, located proximal to the PM, appears to be granular. The outer layer represents at least a part of the peptidoglycan-arabinogalactan polymer [7]. Furthermore, the bacteria posses an additional membrane called mycobacterial outer membrane (MOM). The MOM is mainly composed of long chain mycolic fatty acids (C_60_-C_90_) with free intercalating glycolipids. It is covalently linked to the arabinogalactan-peptidoglycan layer [8] and presents a veritable permeability barrier. The outermost layer of the cell envelope is a capsule composed of polysaccharides, proteins and small amounts of lipids [9].

Protein secretion is essential for all bacteria in order to interact with their environment. In monoderm bacteria export systems that translocate proteins across the PM are sufficient. In diderm bacteria such as the Gram-negatives or mycobacteria secreted proteins have to overcome not only the PM but also the second hydrophobic permeability barrier – the outer membrane. Both the general secretion system (Sec) and the twin-arginine translocation system (Tat) are functional in mycobacteria [10], [11], [12]. Interestingly, it has been shown that mycobacteria possess an accessory, non-essential SecA2 protein (compared to the housekeeping SecA1) which is involved in the export of a specific subset of proteins, e.g. the superoxide dismutase SodA [13]. Furthermore, a high amount of small, highly immunogenic proteins lacking a classical secretion signal peptide has been found in the culture filtrate of *M. tuberculosis* [14]. These proteins have a size of approx. 100 amino acids (aa) and share a Trp-Xaa-Gly (WXG) motif [15]. The most prominent members of this protein family are the early secreted antigen target, 6 kDa (ESAT-6, EsxA) and the culture filtrate protein, 10 kDa (CFP-10, EsxB). Genes coding for WXG-100 family proteins are found in the genome of all mycobacteria and in a wide range of actinobacteria and low G+C content Gram-positives [15]. Most of these WXG-100 proteins are predicted to be exported by a novel type of protein translocation system in mycobacteria often referred to as Type VII secretion system (T7SS) [16] or more general as WXG-100 secretion systems (WSS) [17], [18]. In mycobacteria, where the T7SS have been discovered first, the protein translocation machineries as well as the corresponding genomic regions are commonly referred to as ESAT-6 secretion systems (ESX). This term will be used throughout this article. In *M. tuberculosis* five paralogous ESX regions are annotated (ESX-1 to ESX-5). Several of these ESX regions are also present in other members of the genus *Mycobacterium* [19]. Outside the genus *Mycobacterium*, multiple ESX regions have not been found so far. ESX gene clusters typically also encode proteins of the mycobacterial specific enigmatic PE and PPE families, named after their N-terminal proline-glutamic acid (PE) and proline-proline-glutamic acid (PPE) motifs [20].

RETRACTED

The first ESX protein translocation system found in *M. tuberculosis* (ESX-1) is required for full virulence [21]. Most genes of ESX-1 are located in the region of difference-1 (RD-1), which is prominently absent in the attenuated vaccine strain *Mycobacterium bovis* BCG [22] and in *Mycobacterium microti* [23]. The exact function of ESX-1 and its translocation substrates are not fully understood yet. Among the reported functions are block of phagosome maturation [24], suppression of proinflammatory cytokine production [25] and disruption of membranes [26]. Furthermore, it has been shown that ESX-1 translocation plays an essential role in mycobacterial DNA transfer in *M. smegmatis* [27]. Deletions in the ESX-1 gene cluster seem to increase the donor function, whereas the same deletions abolish reception of transferred DNA. Functional studies on the ESX-2 and ESX-4 systems have not been published so far. Whole genome studies suggest that neither of these two systems is required for *in vitro* growth or virulence [28], [29]. *Mycobacterium leprae* is missing both the ESX-2 and ESX-4 region from its minimal genome [19]. These findings indicate a negligible function of these two ESX clusters. ESX-3 is present in all mycobacterial genomes sequenced so far. In *M. tuberculosis* and in *M. smegmatis* several studies have shown that ESX-3 is involved in iron import [30], [31]. Siegrist *et al.* found evidence, that iron bound to secreted mycobactin can not be utilized in ESX-3 deletion strains [32]. Although *M. smegmatis* tolerates ESX-3 deletions quite well, the system seems to be essential in *M. tuberculosis* since corresponding deletion mutants could not be generated so far [28], [31]. ESX-5 is the phylogenetically youngest ESX region and restricted to slow growing, pathogenic mycobacteria [19]. It has been show to be involved in the secretion of a set of diverse PPE and PE_PGRS proteins [33]. ESX-5 has been linked to virulence in the fish pathogen *M. marinum* [33], [34] and was suggested to play a role in cell death in *M. tuberculosis* related pathogenesis [35].

RETRACTED

The *M. tuberculosis* ESX-1 system (and supposedly the ESX-5 system) is required for full virulence, therefore discovering and characterizing its components is a focal point of mycobacterial virulence research. However, there is a growing interest in the essential ESX-3 system of *M. tuberculosis* [32], [36], [37], [38], [39] since its components represent promising new targets for antimycobacterial drugs. The absence of ESX-protein-translocation reporter limits characterization of ESX systems, especially the identification of components not encoded in the ESX region. In this study we present such a reporter system for studying ESX protein translocation.

## Materials and Methods

### Bacterial strains and growth conditions

*Mycobacterium smegmatis* SMR5, a derivative of *M. smegmatis* mc^2^155, carrying a non-restrictive *rpsL* mutation conferring streptomycin resistance [40] was grown on Middlebrook 7H10 agar supplemented with 10% oleic acid albumin dextrose catalase (OADC, Difco) and in liquid Middlebrook 7H9 supplemented with 10% OADC and with Tween 80 (0.05%) to avoid clumping. When appropriate, antibiotics were added at the following concentrations: ampicillin, 120 µg/ml; streptomycin, 100 µg/ml; hygromycin, 50 µg/ml; kanamycin, 50 µg/ml. The cells were grown at 37°C. Strain designations were as follows: *M. smegmatis* SMR5, *M. smegmatis* Δ*blaS*, a derivative of *M. smegmatis* SMR5 with deleted *blaS* (*MSMEG_2658*) locus and *M. smegmatis* Δ*blaS* Δ*eccD*_3_, a derivative of *M. smegmatis* Δ*blaS* with an additional deletion in *eccD*_3_ (*MSMEG_0623*).

### Plasmids

A series of heterologous fusion protein constructs were cloned and expressed, using the epichromosomal, high copy number shuttle vector pOLYG [41]. All fusion constructs consist of a truncated form of the TEM-1 β-lactamase (‘Bla TEM-1), originally identified in a clinical isolate of *E. coli* [42], and a secreted protein from *M. tuberculosis* or *M. smegmatis*. The truncated form of the β-lactamase (from here on referred to simply as BlaTEM) lacks the N-terminal 19 amino acids (aa) comprising the secretion signal peptide. It is no longer exported on its own. The construction and schematic organization of the reporter constructs is shown in **figure 1**. Unmarked targeted gene deletions were generated using the mycobacterial suicide vector pMCS5 (MobiTec) with an additional hygromycin resistance cassette [43] and a *rpsL* gene [40]. The deleted β-lactamase *blaS* from *M. smegmatis* was complemented *in trans* using the integrative vector pMV361-*blaS*, a derivative of pMV361 [44]. All plasmids used in this study are listed in **table S1 (supporting material)**.

RETRACTED

**Figure 1:** Schematic representation of the reporter fusion constructs. Shown are only the promoter regions, the truncated β-lactamase (*blaTEM*) and the fused ORF with restriction endonuclease sites for cloning (not drawn to scale). Additional epitope tags for anti HA antibodies are also annotated. The roman numbers on the left side correspond to the vector numbers. Along with *blaTEM* the vector pI-blaTEM contains the ORF encoding the 40 aa N-terminal sec-secretion signal peptide of FbpB (Rv1886c). The vector pII-blaTEM originated from pI-blaTEM and contains the additional 285 codons of the mature FbpB. In the plasmid pIII-blaTEM *blaTEM* is C-terminally fused to the ORF *fbpB* (325 codons). In pIV-blaTEM and pV-blaTEM the ORF *esxG* (Rv0287, 96 codons) is either C- or N-terminally fused to *blaTEM*. pVI-blaTEM originates from pIV-blaTEM with *esxG* substituted for *esxB* (*Rv3874*, 99 codons). In pVII-blaTEM and pVIII-blaTEM *esxG* is substituted for either *esxU_mt_* (*Rv3445c, 104 codons*) or *esxU_ms_* (*MSMEG_1538, 102 codons*). 0 stands for pOLYG-*blaTEM* expressing only the truncated version of Bla TEM-1 (267 aa) lacking the 19 aa secretion signal peptide (BlaTEM). Note that the constructs 0 and I-III are expressed by the *fbpB* promoter (368 bp region upstream of the start codon) whereas the *esx* constructs are under the control of the *esxG_mt_* promoter (500 bp region upstream of the start codon).

### Targeted gene replacements

Replacement of the targeted genes in this study - *MSMEG_2658* (*blaS*) and *MSMEG_0623* (*eccD*_3_) - were done by application of the *rpsL* counter selection strategy [40]. Therefore, electrocompetent streptomycin-resistant *M. smegmatis* SMR5 derivatives were transformed with the suicide plasmids pMCS5-*rpsL*-*hyg*-Δ*blaS* and pMCS5-*rpsL*-*hyg*-Δ*eccD*_3_. These vectors carry approx. 1 kbp genomic regions adjacent to the targeted gene and an unmarked deletion in the targeted gene. Transformants were grown on hygromycin containing media and afterwards counter selected using streptomycin. A point mutation in the *rpsL* gene coding for the ribosomal protein S12 renders *M. smegmatis* SMR5 streptomycin resistant. Thus, transformants integrating the knock out plasmid that encodes the *rpsL* ^+^ locus by single cross-over homologous recombination become sensitive to streptomycin again. A second recombination event results in deletion of the target gene (or revision to wild type) and restores the streptomycin resistant and hygromycin sensitive phenotype. The deletion mutant strains were confirmed by Southern blot analysis using specific DNA probes (**Fig. 2**).

RETRACTED

**Figure 2:** Strategy for targeted generation of mutants and Southern blot analysis. (A) Schematic drawing of the *blaS* (*MSMEG_2658*) genomic region of the wild-type and the knock out strain (not drawn to scale). Southern blot analysis confirms the deletion of *blaS* from the genome of *M. smegmatis*. Genomic DNA of *M. smegmatis* was digested with restriction endonuclease *Mlu*I. A DIG labeled PCR fragment from one of the flanking regions was used as a probe. The wild-type band (wt) was calculated to be 3.39 kbp. The 3′ single cross over (sco) bands correspond to lengths of 9.451 kbp and 2.483 kbp, respectively. The knock out strain (Δ) corresponds to a length of 2.483 kbp. (B) Schematic drawing of the *eccD*_3_ (*MSMEG_0623*) genomic region of the wild-type and the knock out strain (not drawn to scale). Southern blot analysis confirms the deletion of *eccD*_3_ from the genome of *M. smegmatis* Δ*blaS*. Genomic DNA was digested with restriction endonuclease *Tth*111I. The wild-type band (wt) was calculated to be 4.309 kbp. The 5′ single cross over (sco) bands correspond to lengths of 10.316 kbp and 4.309 kbp, respectively. The knock out strain (Δ) corresponds to a length of 5.680 kbp.

### Minimal inhibitory concentration (MIC) determination

Broth microdilution tests were performed in a microtiter plate in a total volume of 100 µl. Bacterial strains were pre-cultured in 7H9 broth supplemented with Tween and OADC as described above. Freshly grown cultures were diluted to an OD_600_ of 0.015, and incubated in 7H9 broth in the presence of 2-fold serial dilutions of ampicillin in the range between 400 µg/ml and 0.8 µg/ml. The minimal inhibitory concentration (MIC) is defined as the drug concentration at which no visible growth is observed by eye after an incubation time of 72 h, corresponding to 24 generations.

### Preparation of cell extracts and Western blot analysis

*M. smegmatis* from 10 ml cultures were harvested and resuspended in phosphate-buffered saline (PBS). After a washing step, the cells were disrupted and homogenized by sonication in an ice bath (Elma, Transsonic T460H) for 1–2 hours. Culture filtrate was concentrated using the Amicon Ultra-15 system (Millipore). Proteins were separated by SDS-PAGE (12.5%) and analyzed by Western blot. Antibodies against the β-lactamase were purchased at Antikoerper-online.de.

RETRACTED

## Results

### Targeted inactivation of *blaS* (*MSMEG_2658*)

*M. smegmatis* is naturally resistant to β-lactam antibiotics due to the presence of an exported β-lactamase as demonstrated by Flores *et al.* [45] and confirmed by us (**Tab. 1**). In order to use a β-lactamase as a reporter in *M. smegmatis*, its native major β-lactamase BlaS (MSMEG_2658) had to be disrupted first. The genomic *blaS* was inactivated by targeted gene replacement using the suicide vector pMCS5-*rpsL*-*hyg*-Δ*blaS*. A Southern blot analysis confirming the deletion of *blaS* is shown in **figure 2**. The resulting strain *M. smegmatis* Δ*blaS* was about 16 times more susceptible to ampicillin than the wild-type strain (**Tab. 1**).

### Reporter vectors

Deletion of its native β-lactamase renders *M. smegmatis* Δ*blaS* highly susceptible to ampicillin. This is a prerequisite to use β-lactamases as selectable reporters. We constructed and expressed fusion constructs using the TEM-1 β-lactamase (Bla TEM-1) [42]. Compared to other β-lactamases, Bla TEM-1 has the significant advantage of being compatible with both Sec and Tat signal sequences, because it does not have to be folded prior to its translocation as shown by McCann *et al.* [46]. In order to investigate protein translocation in *M. smegmatis*, particularly ESX-secretion, eight reporter vectors (pI-*blaTEM* to pVIII-*blaTEM*) were constructed. These vectors contain promoters and parts of or entire open reading frames (ORF) of Sec- and ESX-dependent secreted proteins from *M. tuberculosis* (**Fig. 1**). In case of pVIII-*blaTEM* the Esx part (EsxU) of the fusion protein is derived from *M. smegmatis*. The ORF of each secreted protein was ligated in frame with the ORF of *blaTEM* (a truncated version of *bla TEM*-1 without the 19 codons coding the secretion signal peptide). The backbone plasmid for all reporter plasmids was the shuttle vector pOLYG [41]. The vectors were created in a modular design, facilitating the construction of similar constructs as explained in **figure 1**. pOLYG-*blaTEM* expressing only the truncated form of Bla TEM-1 was constructed as a negative control. BlaTEM without additional secretion signal is suspected to be localized in the cytoplasm and therefore not to confer ampicillin resistance.

### Expression of the reporter fusion constructs and ampicillin susceptibility testing in *M. smegmatis* Δ*blaS*

Cell extract and culture supernatant was analyzed for the presence of the reporter protein. Expression of the reporter constructs at the protein level was shown by Western blot analysis with an antibody specific for Bla TEM-1. BlaTEM-1 was readily detected in the cell extracts (**Fig. 3**) but not in the concentrated culture supernatant (data not shown). Ampicillin susceptibility of the β-lactamase (BlaS) knock out strains with or without reporter plasmids was determined by minimal inhibitory concentration (MIC) assays. The results for each strain are shown in **table 1**. All strains were also tested for susceptibility towards hygromycin (resistance conferred by backbone of the pOLYG vectors) and kanamycin (an unrelated antibiotic). The MIC determination shows that all plasmid bearing strains were equally resistant to hygromycin (MIC>500 µg/ml) compared to the not transformed parental strains which were equally susceptible to hygromycin (MIC 20 µg/ml). This suggests a similar reporter plasmid copy number in all strains. All strains – parental and reporter – were found to be equally sensitive to kanamycin (MIC 12.5 µg/ml). Kanamycin binds to the 30S subunit of bacterial ribosomes - an intracellular target (data not shown). Due to the results of the kanamycin resistance determination it is unlikely that the introduced genetic alteration generally heightened the membrane permeability for antibiotics.

RETRACTED

**Figure 3:** Protein expression of BlaTEM reporter constructs shown by Western blot analysis. Fusion-proteins expressed from the nine reporter vectors (pOLYG-*blaTEM* (0) and pI-*blaTEM* to pVIII-*blaTEM*) were separated using SDS-PAGE (12.5% Tris-HCl gels) and blotted onto PVDF membrane. The membrane was incubated with an antibody against the β-lactamase TEM-1. (A) Protein expression of pOLYG-*blaTEM* (calculated mass 31.8 kDa) and the three Sec dependent FbpB β-lactamase fusion-constructs (pI-*blaTEM*, pII-*blaTEM* and pIII-*blaTEM*). Their masses were calculated to be 31.5 kDa, 33.3 kDa, 61.5 kDa and 62.2 kDa, respectively. The apparent molecular weight corresponds to the mass of a mature protein without secretion signal sequence. (B) Expression of β-lactamase fusion products associated with one of the three ESX protein translocation systems in *M. smegmatis* Δ*blaS*: EsxG (ESX-3), EsxB (ESX-1) and EsxU (ESX-4) expressed from pIV-*blaTEM* (40.7 kDa), pVI-*blaTEM* (41.7 kDa), pVII-*blaTEM* (42.3 kDa) and pVIII-*blaTEM* (42.3 kDa). Although the C-terminally fused “EsxG-BlaTEM” (from pV-*blaTEM*; 41.5 kDa) and both ESX-4 associated N-terminally fused “BlaTEM-EsxU” are translated, no ampicillin resistant phenotype could be observed in the MIC assays. As a positve control (+) lysate from *E. coli* expressing Bla TEM-1 from pGEM-T easy (Promega) was used. The negative control (−) consists of lysate resulting from *M. smegmatis* Δ*blaS* with pOLYG.

RETRACTED

**Table 1:** Ampicillin MIC of *M. smegmatis* Δ*blaS* strains with or without reporter plasmid.

strain	plasmid	reporter	MIC (µg/mL) amp
*M. smegmatis* SMR5	none	none	200–400
*M. smegmatis* Δ*blaS*	none	none	12.5–25
*M. smegmatis* Δ*bla*S-*blaS*	pMV361-*blaS* (integrated)	BlaS	200–400
*M. smegmatis* Δ*blaS*	pOLYG-*blaTEM*	BlaTEM	12.5–25
*M. smegmatis* Δ*blaS*	pI-*blaTEM* a	Sec-BlaTEM	100–200
*M. smegmatis* Δ*blaS*	pII-*blaTEM* a	Sec-BlaTEM-‘FbpB	200–400
*M. smegmatis* Δ*blaS*	pIII-*blaTEM* a	FbpB-BlaTEM	200–400
*M. smegmatis* Δ*blaS*	pIV-*blaTEM* b	BlaTEM-EsxG	>400
*M. smegmatis* Δ*blaS*	pV-*blaTEM* b *	EsxG-BlaTEM	12.5–25
*M. smegmatis* Δ*blaS*	pVI-*blaTEM* c	BlaTEM-EsxB	100–200
*M. smegmatis* Δ*blaS*	pVII-*blaTEM* d	BlaTEM-EsxU_Mt_	12.5–25
*M. smegmatis* Δ*blaS*	pVIII-*blaTEM* d	BlaTEM-EsxU_Ms_	12.5–25

Predicted export systems:

a ) Sec,

b ) ESX-3,

c ) ESX-1,

d ) ESX-4.

* Export signal supposedly not recognized since internal.

The MIC data show that the ampicillin sensitive *M. smegmatis* Δ*blaS* strain can be complemented with pMV361-*blaS*, thereby restoring its natural resistance. *M. smegmatis* Δ*blaS* transformed with pOLYG-*blaTEM* (a vector expressing a truncated version of Bla TEM-1 without secretion signal sequence) remains susceptible to ampicillin. Insertion of the Sec signal sequence from the fibronectin binding protein B (Antigen 85B, Rv1886c) FbpB (pI-*blaTEM*) confers ampicillin resistance (MIC 100–200 µg/ml). The resistance is even higher when in addition to the signal peptide the entire FbpB is fused to BlaTEM. The expression cassette: Sec-BlaTEM-FbpB is expressed by pII-*blaTEM* (MIC 200–400 µg/ml). FbpB-BlaTEM is expressed by pIII-*blaTEM* and also confers high level ampicillin resistance (MIC 200–400 µg/ml). These results coincided with results from McCann *et al.* [46].

In order to investigate the functionality of each of the three annotated ESX systems of *M. smegmatis* (ESX-1, ESX-3 and ESX-4) we created a new reporter system by fusing BlaTEM with a *M. tuberculosis* protein supposed to be specific for each system. EsxB (CFP-10, Rv3874) located in the ESX-1 cluster, EsxG (Rv0287) located in the ESX-3 cluster and EsxU (Rv3445c) located in the ESX-4 cluster were chosen. The vector pIV-*blaTEM* expressed fusion protein BlaTEM-EsxG and the vector pV-*blaTEM* the reverse constellation, i.e. EsxG-BlaTEM (**Fig. 1**). pVI-*blaTEM* expressed BlaTEM-EsxB and pVII-*blaTEM* expressed BlaTEM-EsxU. Both pIV-*blaTEM* [BlaTEM-EsxG] and pVI-*blaTEM* [BlaTEM-EsxB] conferred ampicillin resistance in *M. smegmatis* Δ*blaS*. Transformation of the vector pV-*blaTEM* could not confer ampicillin resistance despite expression of the fusion protein (**Fig. 3B**). Vector pVII-*blaTEM* was also unable to confer ampicillin resistance. We hypothesized that the secretion signal of EsxU from *M. tuberculosis* (EsxU_Mt_) was not recognized by *M. smegmatis* ESX-4. Therefore we exchanged EsxU_Mt_ with EsxU from *M. smegmatis* (EsxU_Ms_) (MSMEG_1538) resulting in the reporter vector pVIII-*blaTEM*. Nevertheless, pVIII-*blaTEM* also was not able to confer ampicillin resistance in *M. smegmatis* Δ*blaS* despite expression of the fusion protein (**Fig. 3B**).

RETRACTED

### Targeted inactivation of EccD_3_ (MSMEG_0623) and ampicillin susceptibility testing in *M. smegmatis* Δ*blaS* Δ*eccD*_3_

*EccD*_3_ encodes the supposed pore protein of the ESX-3 secretion system [19]. Using *M. smegmatis* Δ*blaS* as parental strain, a deletion in *eccD*_3_ was generated resulting in strain *M. smegmatis* Δ*blaS* Δ*eccD*_3_. Inactivation of EccD_3_ did not affect susceptibility to ampicillin as compared to the parental strain (**Tab. 2**). A Southern blot confirming the deletion of *eccD*_3_ region is shown in **figure 2**.

The strain deficient in EccD_3_ (*M. smegmatis* Δ*blaS* Δ*eccD*_3_) was transformed with the reporter vectors. Ampicillin susceptibility of *M. smegmatis* Δ*blaS* Δ*eccD*_3_ double knock out strain was determined in the same fashion as in the single knock out strain *M. smegmatis* Δ*blaS*. The results are shown in **table 2**. As expected, the strain expressing the ESX-3 related construct BlaTEM-EsxG was no longer able to confer ampicillin resistance thus confirming the specificity of the reporter construct. Recombinants expressing reporter constructs of the Sec- or ESX-1 pathway were not affected by the deletion of EccD_3_ with respect to the ampicillin resistance phenotype. These results were confirmed by plating the strains on 7H10 Amp (120 µg/ml) and are shown in **figure 4**.

**Figure 4:** Growth of *M. smegmatis* strains on an agar plate containing ampicillin. Freshly grown cultures were diluted to an OD_600_ of 0.015. 1 µl of each strain was streaked in a separate sector on a Middlebrook 7H10 plate containing ampicillin [120 µg/ml]. The plate was incubated for 3 days at 37°C. The parental strain in the sectors 1–5 is *M. smegmatis* Δ*blaS*. The parental strain in sectors 6–8 is *M. smegmatis* Δ*blaS* Δ*eccD_3_*. Additional roman numbers correspond to the reporter vector in each strain (cf. **tables 1** **+** **2**). Reporter constructs: (−): none; 0: *BlaTEM*; II: Sec-BlaTEM-‘FbpB; IV: BlaTEM-EsxG; and VI: BlaTEM-EsxB. Note: The reporter construct BlaTEM-EsxG from pIV-*blaTEM* (sector 7) is no longer able to confer ampicillin resistance when a key component of ESX-3 (EccD_3_) is deleted. In contrast, constructs specific for Sec (sector 6) and ESX-1 (sector 8) dependent translocation still confer an ampicillin resistance phenotype.

RETRACTED

**Table 2:** Ampicillin MIC of *M. smegmatis* Δ*blaS* Δ*eccD*_3_ strains with or without reporter plasmid.

strain	plasmid	reporter	MIC (µg/mL) amp
*M. smegmatis* Δ*blaS* Δ*eccD*_3_	pOLYG-*blaTEM*	BlaTEM	12.5–25
*M. smegmatis* Δ*blaS* Δ*eccD*_3_	pI-*blaTEM* a	Sec-BlaTEM	100–200
*M. smegmatis* Δ*blaS* Δ*eccD*_3_	pII-*blaTEM* a	Sec-BlaTEM-‘FbpB	200–400
*M. smegmatis* Δ*blaS* Δ*eccD*_3_	pIII-*blaTEM* a	FbpB-BlaTEM	200–400
*M. smegmatis* Δ*blaS* Δ*eccD*_3_	pIV-*blaTEM* b	BlaTEM-EsxG	12.5–25
*M. smegmatis* Δ*blaS* Δ*eccD*_3_	pVI-*blaTEM* c	BlaTEM-EsxB	100–200

Predicted export systems:

a ) Sec,

b ) ESX-3,

c ) ESX-1.

## Discussion

In monoderm Gram-positives, protein translocation processes are export processes. In these bacteria, protein export equals protein secretion, since the bacteria do not possess an outer membrane [17]. The majority of protein secretion in monoderm Gram-positives is conducted by the general secretion system (Sec) and the twin arginine transport system (Tat) [38]. In some Gram-positives, protein translocation can also be performed by WXG100-family secretion systems (WSS). WSS are especially found in all diderm Gram-positives, where the Sec, Tat and supposedly WSS are export systems. In mycobacteria, where WSS were described first, the terms type VII secretion system (T7SS) and ESAT-6 secretion systems (ESX) are most commonly used. The substrate translocated by the ESX system is ultimately found in the culture supernatant and thus extracellular. Actual proof that ESX are responsible for one step secretion similar to the Gram-negative type III and type IV secretion systems has yet to be given. A new bioinformatics approach suggests EccB1 and/or EccE1 as MOM channels for ESX-1 substrates [47]. However it is very well possible that an independent, hypothetical translocation machinery is located in the mycobacterial outer membrane handling the second translocation step for all the exported proteins destined for secretion into the extracellular milieu. Much progress has been made in elucidating the mycobacterial protein translocation, however there are still many puzzle pieces missing.

In 2005, Flores *et al.* identified the major secreted β-lactamases of *M. tuberculosis* (BlaC, Rv2068c) and of *M. smegmatis* (BlaS, MSMEG_2658) [48]. The β-lactamase knock out strains were later exploited to investigate protein secretion in *M. tuberculosis* and *M. smegmatis*, respectively. The Tat translocated BlaC [10] and the Sec translocated β-lactamase TEM-1 (Bla TEM-1) [46] - originally identified in a clinical isolate of *E. coli* [42] - were used as reporter in these strains. Bla TEM-1 fulfils all criteria for an export-reporter enzyme. It is small and can easily be fused to other proteins. Bla TEM-1 is inactive in the cytoplasm and can confer ampicillin resistance in a *M. smegmatis* Δ*blaS* strain when exported [46]. For these reasons we used a truncated version of Bla TEM-1 (BlaTEM) – lacking secretion signal peptide – as a reporter in our BlaS knock out strain (*M. smegmatis* Δ*blaS*). The minimal inhibitory concentration (MIC) of ampicillin of *M. smegmatis* Δ*blaS* was about 16-fold lower compared to the wild-type strain. This ampicillin susceptible *M. smegmatis* Δ*blaS* became the parental strain for all other strains. A first series of reporter constructs was generated by C-terminal fusion of the N-terminally truncated Bla TEM-1 (lacking its native secretion signal peptide) to several variants of the fibronectin binding protein B (FbpB; antigen 85b of *M. tuberculosis*). FbpB is secreted via the Sec pathway. Ampicillin resistance was conferred due to expression and export of the heterologous BlaTEM proteins. *M. smegmatis* Δ*blaS* expressing BlaTEM without a signal peptide remained sensitive to ampicillin. These results coincided with results from McCann *et al.* [46].

RETRACTED

We established an ESX-specific reporter system by fusing *blaTEM* N-terminally and in frame with genes encoding proteins associated with the ESX translocation systems such as *esxB* (*cfp*-10, Rv3874), *esxG* (Rv0287) and *esxU* (Rv3445c). The reporter constructs with their suspected translocation machineries are drawn in **figure 5**. The constructs BlaTEM-EsxB and BlaTEM-EsxG conferred ampicillin resistance in *M. smegmatis* Δ*blaS*. EsxB possesses a C-terminal secretion signal sequence [49]. Here we showed that EsxG bears an analogous sequence which is suspected to be specific for ESX-3 protein translocation. The N-terminal fusion-construct EsxG-BlaTEM did not confer ampicillin resistance. Together, these results suggest that the translocation signal sequence has to be located at the C-terminus. Since we could not detect the BlaTEM fusion products in the supernatant using the β-lactamase antibody in Western blots (data not shown), we suspect, that the reporters are exported and remain in the PP. These findings indicate that ESX-dependent secretion comprises two discrete steps, translocation across the PM and subsequently translocation across the MOM. Dissection of these steps is possible since translocation into the PP confers a selectable phenotype. The subsequent translocation step of the reporter constructs may be disturbed because of the heterologous expression, the size of the fusion protein, its folding, or absence of an interaction partner. Interestingly both EsxB and EsxG from *M. tuberculosis* seem to be translocated by *M. smegmatis* without co-expression of the proposed heterodimer partner proteins EsxA_Mt_ and EsxH_Mt_. Eventually EsxB_Mt_ and EsxG_Mt_ can bind to EsxA_Ms_ and EsxH_Ms_ and translocate together. Alternatively, translocation does not require a dimerization step as long as a C-terminal secretion signal is attached to the translocation substrate.

RETRACTED

**Figure 5:** Schematic drawing of the cell envelope and the known protein export systems of *M. smegmatis*. Displayed is a simplified model of a cell envelope (without outer capsular layer) as suggested by cryo-electron tomography images [6], [9]. PM stands for the phospholipid bilayer plasma membrane. The periplasmatic space (PP) contains two electron dense layers of unconfirmed identity L1 and L2. The additional membrane is the mycobacterial outer membrane (MOM). The general secretion system (Sec) is colored brown as is one of its substrate: FbpB. FbpB contains a cleavable Sec signal peptide represented as an attached oval. The twin arginine translocation pathway (Tat) is represented in green. One of its substrate is the mayor secreted β-lactamase BlaS containing a cleavable Tat signal peptide. BlaS is missing in the Δ*blaS* knock out strain. The ESX protein translocation systems 1, 3 and 4 of *M. smegmatis* are drawn together with their suggested heterodimeric substrates: EsxA/B, EsxH/G and EsxT/U. EsxB, EsxG and EsxU posses a C-terminal secretion signal represented as a small attached circle. All reporter constructs used in this study are schematically represented and lettered with the corresponding roman number (cf. **Fig. 1**). The β-lactamase BlaTEM fusion partner is represented as a red box (Bla). Solid arrows indicate a functional translocation event, dotted arrow indicate that translocation function has not been demonstrated so far. The grey oval with the question mark drawn in the MOM represents a yet unknown translocation system for crossing the second permeability barrier.

To test specificity of the ESX system for translocation reporters we created an ESX-3 deletion strain (*eccD*_3_, *MSMEG_0623*) of *M. smegmatis* Δ*blaS*. BlaTEM-EsxG was no longer able to confer ampicillin resistance in *M. smegmatis* Δ*blaS* Δ*eccD*_3_, indicating that EsxG is specifically translocated by ESX-3. In contrast Sec- and ESX-1 reporter constructs still conferred an ampicillin resistance phenotype. This indicates that other translocation systems are not affected by EccD_3_ deletion.

RETRACTED

BlaTEM-EsxU was unable to confer ampicillin resistance even though it was expressed. To test if merely the homology between the secretion signal of EsxU_Mt_ (Rv3445c) and EsxU_Ms_ (MSMEG_1538) was too low, the two genes were exchanged in the BlaTEM constructs. Nonetheless BlaTEM-EsxU_Ms_ was not able to confer ampicillin resistance in *M. smegmatis* Δ*blaS*. EsxU was never found in culture filtrates of *M. tuberculosis* [50] and also does not seem to be exported in our experiments. Therefore, we speculate that ESX-4 in both *M. tuberculosis* and in *M. smegmatis* is either not transcribed or not functional as a translocation system anymore. The absence of the genes coding for an AAA+ ATPase (EccA) and the transmembrane protein (EccE) in the ESX-4 operon supports the latter hypothesis. Also missing are genes coding for PE and PPE proteins.

In conclusion we have established a reporter system for functional investigation of ESX protein translocation. The reporter system works with both ESX-1 and ESX-3 substrates. Since ESX-3 is essential in *M. tuberculosis* but not in *M. smegmatis*, we have now an excellent format for studying components of ESX-3 dependent protein translocation. The reporter system facilitates identification and confirmation of novel components of ESX protein translocation systems for plasma membrane transport by a genetic approach. Furthermore, we have for the first time a tool for high throughput screening of drugs interfering with crucial components of the ESX system (ESX-1 or ESX-3), which could give us a new edge in fighting drug resistant *M. tuberculosis* strains as proposed by Feltcher *et al.* [38].

## Supporting Information

Table S1 **Plasmids used in this study.**
(DOC)

## References

[1] Brosch R, Gordon SV, Marmiesse M, Brodin P, Buchrieser C (2002). A new evolutionary scenario for the Mycobacterium tuberculosis complex.. Proc Natl Acad Sci U S A.

[2] Clark-Curtiss JE, Haydel SE (2003). Molecular genetics of Mycobacterium tuberculosis pathogenesis.. Annu Rev Microbiol.

[3] Rohde K, Yates RM, Purdy GE, Russell DG (2007). Mycobacterium tuberculosis and the environment within the phagosome.. Immunol Rev.

[4] McLaughlin B, Chon JS, MacGurn JA, Carlsson F, Cheng TL (2007). A mycobacterium ESX-1-secreted virulence factor with unique requirements for export.. PLoS Pathog.

[5] Torrelles JB, Schlesinger LS (2010). Diversity in Mycobacterium tuberculosis mannosylated cell wall determinants impacts adaptation to the host.. Tuberculosis (Edinb).

[6] Hoffmann C, Leis A, Niederweis M, Plitzko JM, Engelhardt H (2008). Disclosure of the mycobacterial outer membrane: cryo-electron tomography and vitreous sections reveal the lipid bilayer structure.. Proc Natl Acad Sci U S A.

RETRACTED

[7] Zuber B, Chami M, Houssin C, Dubochet J, Griffiths G (2008). Direct visualization of the outer membrane of mycobacteria and corynebacteria in their native state.. J Bacteriol.

[8] Nikaido H, Kim SH, Rosenberg EY (1993). Physical organization of lipids in the cell wall of Mycobacterium chelonae.. Mol Microbiol.

[9] Sani M, Houben EN, Geurtsen J, Pierson J, de Punder K (2010). Direct visualization by cryo-EM of the mycobacterial capsular layer: a labile structure containing ESX-1-secreted proteins.. PLoS Pathog.

[10] McDonough JA, McCann JR, Tekippe EM, Silverman JS, Rigel NW (2008). Identification of functional Tat signal sequences in Mycobacterium tuberculosis proteins.. J Bacteriol.

[11] Cole ST, Brosch R, Parkhill J, Garnier T, Churcher C (1998). Deciphering the biology of Mycobacterium tuberculosis from the complete genome sequence.. Nature.

[12] Wiker HG, Wilson MA, Schoolnik GK (2000). Extracytoplasmic proteins of Mycobacterium tuberculosis - mature secreted proteins often start with aspartic acid and proline.. Microbiology.

[13] Braunstein M, Espinosa BJ, Chan J, Belisle JT, Jacobs WR (2003). SecA2 functions in the secretion of superoxide dismutase A and in the virulence of Mycobacterium tuberculosis.. Mol Microbiol.

[14] Sorensen AL, Nagai S, Houen G, Andersen P, Andersen AB (1995). Purification and characterization of a low-molecular-mass T-cell antigen secreted by Mycobacterium tuberculosis.. Infect Immun.

[15] Pallen MJ (2002). The ESAT-6/WXG100 superfamily – and a new Gram-positive secretion system?. Trends Microbiol.

[16] Abdallah AM, Gey van Pittius NC, Champion PA, Cox J, Luirink J (2007). Type VII secretion–mycobacteria show the way.. Nat Rev Microbiol.

[17] Desvaux M, Hebraud M, Talon R, Henderson IR (2009). Secretion and subcellular localizations of bacterial proteins: a semantic awareness issue.. Trends Microbiol.

[18] Sutcliffe IC (2010). New insights into the distribution of WXG100 protein secretion systems.. Antonie Van Leeuwenhoek.

[19] Gey Van Pittius NC, Gamieldien J, Hide W, Brown GD, Siezen RJ (2001). The ESAT-6 gene cluster of Mycobacterium tuberculosis and other high G+C Gram-positive bacteria.. Genome Biol.

[20] Gey van Pittius NC, Sampson SL, Lee H, Kim Y, van Helden PD (2006). Evolution and expansion of the Mycobacterium tuberculosis PE and PPE multigene families and their association with the duplication of the ESAT-6 (esx) gene cluster regions.. BMC Evol Biol.

[21] Lewis KN, Liao R, Guinn KM, Hickey MJ, Smith S (2003). Deletion of RD1 from Mycobacterium tuberculosis mimics bacille Calmette-Guerin attenuation.. J Infect Dis.

RETRACTED

[22] Ganguly N, Siddiqui I, Sharma P (2008). Role of M. tuberculosis RD-1 region encoded secretory proteins in protective response and virulence.. Tuberculosis (Edinb).

[23] Brodin P, Eiglmeier K, Marmiesse M, Billault A, Garnier T (2002). Bacterial artificial chromosome-based comparative genomic analysis identifies Mycobacterium microti as a natural ESAT-6 deletion mutant.. Infect Immun.

[24] Xu J, Laine O, Masciocchi M, Manoranjan J, Smith J (2007). A unique Mycobacterium ESX-1 protein co-secretes with CFP-10/ESAT-6 and is necessary for inhibiting phagosome maturation.. Mol Microbiol.

[25] Stanley SA, Raghavan S, Hwang WW, Cox JS (2003). Acute infection and macrophage subversion by Mycobacterium tuberculosis require a specialized secretion system.. Proc Natl Acad Sci U S A.

[26] de Jonge MI, Pehau-Arnaudet G, Fretz MM, Romain F, Bottai D (2007). ESAT-6 from Mycobacterium tuberculosis dissociates from its putative chaperone CFP-10 under acidic conditions and exhibits membrane-lysing activity.. J Bacteriol.

[27] Coros A, Callahan B, Battaglioli E, Derbyshire KM (2008). The specialized secretory apparatus ESX-1 is essential for DNA transfer in Mycobacterium smegmatis.. Mol Microbiol.

[28] Sassetti CM, Boyd DH, Rubin EJ (2003). Genes required for mycobacterial growth defined by high density mutagenesis.. Mol Microbiol.

[29] Sassetti CM, Rubin EJ (2003). Genetic requirements for mycobacterial survival during infection.. Proc Natl Acad Sci U S A.

[30] Maciag A, Piazza A, Riccardi G, Milano A (2009). Transcriptional analysis of ESAT-6 cluster 3 in Mycobacterium smegmatis.. BMC Microbiol.

[31] Serafini A, Boldrin F, Palu G, Manganelli R (2009). Characterization of a Mycobacterium tuberculosis ESX-3 conditional mutant: essentiality and rescue by iron and zinc.. J Bacteriol.

[32] Siegrist MS, Unnikrishnan M, McConnell MJ, Borowsky M, Cheng TY (2009). Mycobacterial Esx-3 is required for mycobactin-mediated iron acquisition.. Proc Natl Acad Sci U S A.

[33] Abdallah AM, Verboom T, Weerdenburg EM, Gey van Pittius NC, Mahasha PW (2009). PPE and PE_PGRS proteins of Mycobacterium marinum are transported via the type VII secretion system ESX-5.. Mol Microbiol.

[34] Abdallah AM, Verboom T, Hannes F, Safi M, Strong M (2006). A specific secretion system mediates PPE41 transport in pathogenic mycobacteria.. Mol Microbiol.

[35] Abdallah AM, Bestebroer J, Savage ND, de Punder K, van Zon M (2011). Mycobacterial Secretion Systems ESX-1 and ESX-5 Play Distinct Roles in Host Cell Death and Inflammasome Activation.. J Immunol.

[36] Ilghari D, Lightbody KL, Veverka V, Waters LC, Muskett FW (2011). Solution structure of the Mycobacterium tuberculosis EsxG.EsxH complex: functional implications and comparisons with other M. tuberculosis Esx family complexes.. J Biol Chem.

RETRACTED

[37] Arbing MA, Kaufmann M, Phan T, Chan S, Cascio D (2010). The crystal structure of the Mycobacterium tuberculosis Rv3019c-Rv3020c ESX complex reveals a domain-swapped heterotetramer.. Protein Sci.

[38] Feltcher ME, Sullivan JT, Braunstein M (2011). Protein export systems of Mycobacterium tuberculosis: novel targets for drug development?. Future Microbiol.

[39] Sweeney KA, Dao DN, Goldberg MF, Hsu T, Venkataswamy MM (2011). A recombinant Mycobacterium smegmatis induces potent bactericidal immunity against Mycobacterium tuberculosis.

[40] Sander P, Meier A, Bottger EC (1995). rpsL+: a dominant selectable marker for gene replacement in mycobacteria.. Mol Microbiol.

[41] O'Gaora P, Barnini S, Hayward C, Filley E, Rook G (1997). Mycobacteria as immunogens: development of expression vectors for use in multiple mycobacterial species.. Med Princ Prac.

[42] Datta N, Kontomichalou P (1965). Penicillinase synthesis controlled by infectious R factors in Enterobacteriaceae.. Nature.

[43] Wanner RM, Castor D, Guthlein C, Bottger EC, Springer B (2009). The uracil DNA glycosylase UdgB of Mycobacterium smegmatis protects the organism from the mutagenic effects of cytosine and adenine deamination.. J Bacteriol.

[44] Stover CK, de la Cruz VF, Fuerst TR, Burlein JE, Benson LA (1991). New use of BCG for recombinant vaccines.. Nature.

[45] Flores AR, Parsons LM, Pavelka MS (2005). Genetic analysis of the beta-lactamases of Mycobacterium tuberculosis and Mycobacterium smegmatis and susceptibility to beta-lactam antibiotics.. Microbiology.

[46] McCann JR, McDonough JA, Pavelka MS, Braunstein M (2007). Beta-lactamase can function as a reporter of bacterial protein export during Mycobacterium tuberculosis infection of host cells.. Microbiology.

[47] Das C, Ghosh TS, Mande SS (2011). Computational Analysis of the ESX-1 Region of Mycobacterium tuberculosis: Insights into the Mechanism of Type VII Secretion System.. PLoS One.

[48] Flores AR, Parsons LM, Pavelka MS (2005). Characterization of novel Mycobacterium tuberculosis and Mycobacterium smegmatis mutants hypersusceptible to beta-lactam antibiotics.. J Bacteriol.

[49] Champion PA, Stanley SA, Champion MM, Brown EJ, Cox JS (2006). C-terminal signal sequence promotes virulence factor secretion in Mycobacterium tuberculosis.. Science.

[50] Malen H, Berven FS, Fladmark KE, Wiker HG (2007). Comprehensive analysis of exported proteins from Mycobacterium tuberculosis H37Rv.. Proteomics.

